This article has been retracted.

# Long-term load duration induces N-cadherin down-regulation and loss of cell phenotype of nucleus pulposus cells in a disc bioreactor culture

**DOI:** 10.1042/BSR20160582

**Published:** 2017-04-28

**Authors:** Pei Li, Ruijie Zhang, Liyuan Wang, Yibo Gan, Yuan Xu, Lei Song, Lei Luo, Chen Zhao, Chengmin Zhang, Bin Ouyang, Bing Tu, Qiang Zhou

**Affiliations:** 1 Department of Orthopedic Surgery, Southwest Hospital, Third Military Medical University, Chongqing 400038, China; 2 Department of Respiratory Medicine, The Third Xiangya Hospital, Central South University, Changsha, Hunan 410013, China; 3 Department of Orthopedic Surgery, Xinqiao Hospital, Third Military Medical University, Chongqing 400038, China

**Keywords:** compression, degeneration, nucleus pulposus, N-cadherin, organ culture

## Abstract

Long-term exposure to a mechanical load causes degenerative changes in the disc nucleus pulposus (NP) tissue. A previous study demonstrated that N-cadherin (N-CDH)-mediated signalling can preserve the NP cell phenotype. However, N-CDH expression and the resulting phenotype alteration in NP cells under mechanical compression remain unclear. The present study investigated the effects of the compressive duration on N-CDH expression and on the phenotype of NP cells in an *ex vivo* disc organ culture. Porcine discs were organ cultured in a self-developed mechanically active bioreactor for 7 days. The discs were subjected to different dynamic compression durations (1 and 8 h at a magnitude of 0.4 MPa and frequency of 1.0 Hz) once per day. Discs that were not compressed were used as controls. The results showed that long-term compression duration (8 h) significantly down-regulated the expression of N-CDH and NP-specific molecule markers (Brachyury, Laminin, Glypican-3 and Keratin 19), attenuated Alcian Blue staining intensity, decreased glycosaminoglycan (GAG) and hydroxyproline (HYP) contents and decreased matrix macromolecule (aggrecan and collagen II) expression compared with the short-term compression duration (1 h). Taken together, these findings demonstrate that long-term load duration can induce N-CDH down-regulation, loss of normal cell phenotype and result in attenuation of NP-related matrix synthesis in NP cells.

## Introduction

In the past several decades, intervertebral disc degeneration (IDD) has become a widely discussed topic among orthopaedic surgeons [1–3]. IDD can lead to back and leg pain in patients and cause a heavy economic burden on the social healthcare system. Despite increasing progression in the field of intervertebral disc research, further studies are needed to uncover the pathogenesis of disc degeneration to develop effective treatments.

Mechanical load is regarded as a potential risk factor for initiating and/or aggravating the disc degeneration process [4,5]. To verify this point, many research teams around the world have carried out multiple studies. A consensus of previous studies is that mechanical overload and long-term mechanical load have a harmful influence on healthy disc biology [6–8]. Consistent with this idea, people who are engaged in heavy manual labour are prone to degenerative disc disease [9]. At the cellular and molecular levels, our studies and the studies of others, have indicated that an unphysiological mechanical load causes catabolic matrix remodelling in disc nucleus pulposus (NP) region [10–14]. Since a stable cell phenotype is necessary for maintaining normal cell function, including cellular matrix synthesis bioactivity [15,16], the alteration of the NP cell phenotype may contribute to an attenuated NP matrix homoeostasis under an unphysiological mechanical load.

N-cadherin (N-CDH) is a calcium-dependent adhesion molecule that has been suggested to play an important role in the development of neural crest and the formation of neuronal connections [17,18]. In the past few years, several studies have revealed that N-CDH is highly expressed in healthy and normal disc NP cells compared with degenerative NP cells, adjacent disc annulus fibrosus (AF) cells and cartilage endplate (CEP) cells [19,20]. In addition, an *in vitro* functional study has demonstrated that N-CDH-mediated signalling is helpful in maintaining a normal juvenile NP phenotype and in NP matrix synthesis *in vitro* [21,22]. When considering the positive effects of N-CDH on the normal NP cell phenotype and the negative effects of the unphysiological load on NP matrix remodelling, we suggest that attenuation of N-CDH-mediated signalling may be partly responsible for the mechanical load induced degenerative changes in the disc NP region. However, no study yet has reported expression changes of N-CDH and the resulting NP cell phenotype alteration under a mechanical load.

Therefore, we investigated N-CDH expression and NP cell phenotype alterations under different mechanical compression durations. Because disc organ culture can be performed at a near physiological condition due to its ability to maintain the structural integrity and normal extracellular environment of disc cells [23–25], we used an *ex vivo* disc bioreactor culture system in the present study, which has been implemented previously.

## Materials and methods

### Ethical statement

The experimental pigs (3–4 months old) were purchased from the Animal Center of Third Military Medical University, Chongqing, China. The present study complied with the guidelines and regulations of the Ethics Committee at Southwest Hospital affiliated to the Third Military Medical University.

### Porcine disc harvest and bioreactor culture

Porcine discs (T11-L5) containing the CEP were separated under sterile conditions as described recently [10]. To protect the integrity of disc structure, a dissecting microscope was used to further remove the vertebral bones. After the disc area (Area≈ττ (W_ap_W_lat_)/4, where the W_ap_ and W_lat_ are the anterior-posterior and lateral widths respectively) was measured to calculate the compressive magnitude [26], the discs were organ cultured for 7 days using our self-developed bioreactor (Figure 1). The viability of the disc tissues within this bioreactor culture system has been verified recently [27]. The discs were assigned to different compression duration groups (1 or 8 h per day at a magnitude of 0.4 MPa and frequency of 1.0 Hz). The discs without compression were used as controls. The compression durations (1 and 8 h) were chosen because they are within the human physiological condition in terms of people working 8 h a day. Because a recent study demonstrated that 0.4 MPa is a healthy compressive magnitude [28], which is also the physiological disc pressure for a person in the upright position [29]), we chose 0.4 MPa as our compressive magnitude to minimize damage interference to the disc NP tissue caused by the compressive magnitude. All discs were cultured in DMEM/F12 culture medium (HyClone, U.S.A.), which was supplemented with 10% (v/v) FBS (Gibco, U.S.A.) and 1% (v/v) penicillin-streptomycin (Gibco, U.S.A.). Due to the discrepancy between different vertebrae levels, discs from the same levels were used for the same assay. For example, the immunohistochemistry staining assay was performed on the same three discs (L1/2, L2/3 and L3/4) from different animals.

**Figure 1:** Schematic of bioreactor system used in the present study (**A**) Overview photograph of the bioreactor platform. (**B**) Primary units of the bioreactor system ((a) tissue-culture chamber; (b) peristaltic pump; (c) medium reservoir)).

### Alcian Blue staining assay

After 7 days of organ culture, all discs were sequentially fixed with 4% paraformaldehyde for 48 h, decalcified with 10% EDTA for 15–18 days and embedded in paraffin. Then, 5 μm-thick cross-sections were prepared and stained with an Alcian Blue solution to observe the proteoglycan (PG) distribution in the NP tissue. All sections were observed under light microscope (Olympus BX51). The staining intensity (IOD) was analysed using the Image-Pro Plus software (Version 5.1, Media Cybernetics, Inc.) and it was used for comparison among groups.

### RT-PCR analysis

RT-PCR was performed to analyse mRNA expression of target genes. The total RNA was extracted with TRIzol reagent (Invitrogen, U.S.A.) according to the manufacturer’s instructions. In total, 1 μg RNA in each group was reverse transcribed using a Reverse Transcription Kit (Roche, Switzerland). A system, which included primers (Table 1), cDNA samples and Taq PCR MasterMix (TIANGEN, China), was used to perform RT-PCR. GAPDH and β-actin were used as reference genes. Finally, the PCR products were separated by electrophoresis on a 2.5% agarose gel and visualized by staining with GoldView Nucleic acid dye (Biohao, China). The DNA bands were analysed using the ImageJ software (National Institute of Health, U.S.A.) to calculate the respective grey values that were used to for comparison among groups. For the statistical analysis, expression of target genes was normalized to the mean expression of reference genes (GAPDH and β-actin).

**Table 1:** Primers of target genes

Gene	Source	Accession number	Forward (5′-3′)	Reverse (5′-3′)
*GAPDH*	Pig	NM_001206359.1	ACCTCCACTACATGGTCTACA	ATGACAAGCTTCCCGTTCTC
*β-actin*	Pig	XM_003124280.4	AGAGCAAGAGAGGCATCCTG	CACGCAGCTCGTTGTAGAAG
*Aggrecan*	Pig	NM_001164652.1	CGTGGTCCAGCACTTCTAAA	AGTCCACTGAGATCCTCTACTC
*Collagen II*	Pig	XM_001925959.4	CCGGGTGAACGTGGAGAGACTG	CGCCCCCACAGTGCCCTC
*N-CDH*	Pig	XM_013996117.1	AACAGCAACGACGGCTTAGT	GACTGAGGTGGGTGCTGAAT
*Brachyury*	Pig	XM_001928144.4	GCCTCGAATCCACATCGTGA	TCACCGCTATGAACTGGGTC
*Laminin*	Pig	XM_005667736.2	ACGTGGTTGGAAGAAAGTGC	GACGGGATCACAGAAAGCAT
*Glypican-3*	Pig	XM_013986449.1	TGCCAAGAACTACACCAACG	TCCGAACCCAGGATGTAGAG
*PTN*	Pig	NM_214336.1	CCCATTCTCCATTTCCCTTC	TGGCTTTTCCTCTGCTCTTC
*Keratin 19*	Pig	XM_003131437.3	GGCAGAACCAGGAGTACCAG	GCCTTGATGATGGTCAGGTT

### Immunohistochemistry staining

Immunohistochemistry staining was performed as previously described [10]. Briefly, after dewaxing, antigen retrieval and inactivation of endogeneous peroxidase, the disc sections were incubated with primary antibodies against aggrecan (Novus, NB120-11570, diluted 1:200) and collagen II (Abcam, ab34712, diluted 1:200) overnight at 4°C. This was followed by incubation with corresponding HRP–conjugated secondary antibodies for 2 h at 37°C. After colour development with diaminobenzidine (DAB), all sections were observed under light microscope (Olympus BX51). The staining intensity (IOD) was analysed using the Image-Pro Plus software (Version 5.1, Media Cybernetics, Inc.), and it was used for comparison among groups.

### Western blotting assay

The protein expression of N-CDH was analysed by Western blotting. Briefly, the total protein was extracted from isolated porcine disc NP tissue using RIPA solution (Beyotime, China). The protein samples were subjected to SDS/PAGE electrophoresis and transferred on to PVDF membranes. After membranes were incubated with primary antibodies (N-CDH, Abcam, ab18203, diluted 1:1000; β-actin, Proteintech, 60008-1-Ig, diluted 1:2000) at 4°C overnight and the corresponding secondary antibodies (ZSGB-BIO, China, diluted 1:2000) at 37°C for 2 h, the protein bands were developed using a SuperSignal West Pico Trial Kit (Thermo, U.S.A.). After the grey values of protein bands were analysed using ImageJ software (National Institutes of Health, U.S.A.), the protein expression of N-CDH was normalized to that of β-actin. In addition, the protein bands transferred on to the PVDF membrane were visualized by Ponceau staining.

### Biochemical content measurement

After 7 days of organ culture, porcine disc NP tissues were isolated for the quantification of glycosaminoglycan (GAG) and hydroxyproline (HYP). Briefly, NP tissues used for GAG content measurement were lyophilized for 24 h and digested with papain for 24 h at 60°C. The GAG content was determined according to the standard curve created by gradient concentrations of shark cartilage chondroitin sulfate using the dimethyl Methylene Blue (DMMB) method [30]. The HYP content was analysed using a HYP quantification kit (Nanjing Jiancheng, China) according to the manufacturer’s instructions.

### Statistics

All numerical data in the present study were expressed as the mean ± S.D. and analysed using SPSS 13.0 software. Each experiment was performed in triplicate. After a homogeneity test for variance was completed, one-way ANOVA was performed, which was followed by an LSD post hoc test. A significant difference was indicated when the *P*-value<0.05.

## Results

### Long-term load duration decreased N-CDH expression in porcine disc NP cells

Because it is very difficult to obtain adequate intact human disc samples in clinical practice, an *ex* *vivo* porcine disc bioreactor culture system was adopted to study the response of N-CDH expression to different compression durations. The results showed that both the gene and the protein expression of N-CDH were significantly down-regulated in the long-term load duration (8 h per day) group compared with that in the short-term load duration (1 h per day) group and that in the control group. Moreover, N-CDH expression in the short-term load duration group was similar to that in the control group (Figure 2). These findings indicate that a long-term load duration can lead to a decrease in N-CDH expression.

**Figure 2:** Long-term load duration decreased N-CDH expression in porcine disc NP cells (**A**) RT-PCR analysis of N-CDH gene expression. GAPDH and β-actin were used as reference genes. Gene expression of N-CDH was normalized to the mean expression of GAPDH and β-actin. (**B**) Western blotting analysis of N-CDH protein expression and photographs of Ponceau staining of protein bands on the PVDF membrane. The results showed that long-term load duration (8 h) significantly decreased N-CDH expression level compared with the short-term load duration (1 h) and the control (non-compression) both at gene and protein levels. Data are expressed as the means ± S.D., *n*=3. ^#^: indicates a significant difference (*P*<0.05) when compared with the control group. *: indicates a significant difference between two groups (*P*<0.05).

### Long-term load duration down-regulated gene expression of NP cell-specific markers in porcine disc NP cells

Loss of a normal NP cell phenotype is widely reported during disc degeneration. An attenuated normal NP cell phenotype may cause abnormal cellular biological functions including matrix biosynthesis [15,16]. In the present study, we also evaluated changes in NP-specific marker expression under different compression durations. The results showed that the expression of all the selected NP markers, except PTN, was significantly down-regulated in the long-term load duration (8 h per day) group compared with that in the short-term load duration (1 h per day) group and that in the control group. However, no significant difference for these NP-specific markers was found between the control group and the short-term load duration group (Figure 3). This indicates that a long-term compression duration is not beneficial for maintenance of the normal NP cell phenotype.

**Figure 3:** Long-term load duration down-regulated gene expression of NP cell-specific markers in porcine disc NP cells An RT-PCR assay was used to investigate NP cell-specific marker expression under different compression durations (1 or 8 h per day). GAPDH and β-actin were used as reference genes. Gene expression of target genes was normalized to the mean expression of GAPDH and β-actin. The results showed that long-term load duration (8 h per day) significantly decreased expression of all selected NP markers except PTN compared with the short-term load duration (1 hour per day) and the control (non-compression). Data are expressed as the means ± SD, *n*=3. ^#^: indicates a significant difference (*P*<0.05) when compared with the control group. *: indicates significant difference between two groups (*P*<0.05).

### Long-term load duration decreased expression of NP matrix macromolecules in porcine disc NP cells

Aggrecan and collagen II are the main components of the NP matrix. During disc degeneration, the degenerative changes first occur in the NP region. Such changes include a decreased PG content and a transition of type II collagen to type I collagen [31]. In the present study, we also found that gene expression and protein deposition of matrix macromolecules (aggrecan and collagen II) were decreased in the long-term load duration (8 h per day) group compared with that in the short-term load duration (1 h per day) group, which were indicated by the RT-PCR assay (Figure 4A) and the immunohistochemistry assay (Figure 4B). However, expression of aggrecan and collagen II in the short-term load duration (1 h per day) group was increased compared with that in the control group. This confirms that long-term exposure to mechanical load can induce degenerative changes in the disc matrix.

**Figure 4:** Long-term load duration decreased expression of NP matrix macromolecules in porcine disc NP cells (**A**) RT-PCR analysis of gene expression of aggrecan and collagen II. GAPDH and β-actin were used as reference genes. Gene expression of target genes was normalized to the mean expression of GAPDH and β-actin. (**B**) Immunohistochemistry staining of aggrecan and collagen II. Magnification: 200×, scale =100 μm. The results showed that long-term load duration (8 h per day) significantly decreased gene expression of matrix molecules (aggrecan and collagen II) and their protein deposition within the NP tissue compared with the short-term load duration (1 h per day) and the control (non-compression). Data are expressed as the means ± S.D., *n*=3. ^#^: indicates a significant difference (*P*<0.05) when compared with the control group. *: indicates a significant difference between two groups (*P*<0.05).

### Long-term load duration decreased matrix component content in porcine disc NP cells

To further verify the effects of compression duration on disc NP matrix components, we performed an Alcian Blue assay to observe the PG distribution within the disc NP region and performed biochemical assays to analyse the GAG and HYP contents. The results showed that Alcian Blue staining intensity was lower in the long-term compression duration (8 h per day) group than that in the short-term (1 h per day) group, indicating that the PG content in the long-term compression duration group is decreased (Figure 5A). In addition, long-term compression duration (8 h per day) also significantly decreased the GAG and HYP contents within NP tissue compared with that in the short-term compression duration (1 h per day) (Figure 5B). Taken together, these results further indicate that long-term compression duration can inhibit disc NP matrix synthesis.

**Figure 5:** Long-term load duration decreased matrix component content in porcine disc NP cells (**A**) Alcian Blue staining of PG content within the porcine disc NP tissue. Magnification: 200×, scale =100 μm. (**B**) GAG and HYP contents of porcine disc NP tissue. The results showed that long-term load duration (8 h per day) significantly decreased gene expression of matrix molecules (aggrecan and collagen II) and their protein deposition within the NP tissue compared with the short-term load duration (1 h per day) and the control (non-compression). Data are expressed as the means ± S.D., *n*=3. ^#^: indicates a significant difference (*P*<0.05) when compared with the control group. *: indicates a significant difference between two groups (*P*<0.05).

## Discussion

An altered phenotype is a classical phenomenon in degenerative disc NP cells [16,32–35]. Mechanical load plays an important regulatory role in the disc degeneration process [4,5]. However, the effects of compression duration on the NP cell phenotype remain incompletely studied. N-CDH is reported to be important in maintaining a normal NP cell phenotype [21,22]. Our study demonstrated that the long-term compression duration (8 h per day) could simultaneously decrease the expression of N-CDH and NP-specific markers and induce degenerative changes of disc NP matrix in the porcine disc organ culture. These results partly provide a clue to the relationship between N-CDH expression, NP cell phenotype and NP matrix homoeostasis under long-term mechanical compression.

Although N-CDH was first found to be involved in the development of neural crest and formation of neuronal connections [17,18], recent studies have identified N-CDH expression in disc NP tissue [21,22]. More importantly, a review paper demonstrated that N-CDH is a specific molecule that distinguishes normal NP cells from degenerate NP cells, disc AF cells and disc cartilage CEP cells [12]. Furthermore, a recent study showed that N-CDH-mediated signalling can maintain expression of specific markers (Brachyury and Laminin 1) of juvenile NP cells [21]. Additionally, inhibition of N-CDH-mediated signalling could induce changes associated with disc degeneration, including down-regulation of NP matrix molecules (aggrecan and collagen II) and a decrease in GAG content [21,22]. Based on these findings, those studies concluded that N-CDH could control both NP cell phenotype and matrix biosynthesis, which are important in preservation of healthy disc NP tissues.

Similar to numerous previous studies [36,37], we found a long-term load duration decreased the macromolecule (aggrecan and collagen II) expression and matrix biochemical content (GAG and HYP). Furthermore, the expression of specific markers in juvenile NP cells was also down-regulated in the long-term load duration group. These findings confirm that the long-term exposure to mechanical compression is not helpful for maintaining the healthy status of disc NP cells. In the present study, using the *ex vivo* porcine disc organ culture, we first reported that a long-term load duration could decrease N-CDH expression in NP cells compared with a short-term load duration. Based on the previously reported protective effects of N-CDH on expression of NP cell-specific markers and NP matrix synthesis, these findings indicate that attenuation of N-CDH-mediated signalling may be partly responsible for mechanical load-induced degenerative changes in the disc NP region. However, N-CDH knockdown and N-CDH overexpression experiments are needed to verify this idea and explore the potential molecular mechanisms in the future.

On the other hand, our study showed that NP matrix biosynthesis was maintained in the short-term load duration group compared with that in the control group. This result is similar to the results of recent study [10]. Moreover, N-CDH expression and expression of several NP cell-specific markers were also similar between the control group and the short-term load duration group. Considering the positive effects of N-CDH on preserving the NP cell phenotype [21,22], we conclude that promotion of NP matrix biosynthesis in the short-term load duration group is caused by maintenance of N-CDH expression, which keeps the normal NP cell phenotype.

The present study has several limitations. First, this is a descriptive investigation and the underlying mechanisms were not explored. Second, though porcine discs were used to study disc biology in many studies [38–40], results in the present study may have limited stringency in reproducing the mechanobiology of the adult disc because of the high content of notochordal cells in the immature porcine disc. Third, although we drew conclusions by considering previous findings, activation and/or inhibition experiments were not performed to verify the role of N-CDH in regulating the NP cell phenotype and resulting NP matrix biosynthesis under different compression durations. In future studies, we will verify the effects of N-CDH expression on NP cell phenotype by performing N-CDH overexpression and knockdown experiments.

We demonstrate that N-CDH down-regulation coincides with the down-regulation in the expression of NP cell-specific markers and a decrease in NP matrix biosynthesis under long-term compression duration. When considering the reported protective effects of N-CDH on the NP cell phenotype and NP matrix biosynthesis, our findings indirectly suggest that N-CDH down-regulation may contribute to the NP cell phenotype alteration and the NP matrix degenerative changes under long-term compression duration.

## Abbreviations

AF: annulus fibrosus
CEP: cartilage endplate
GAG: glycosaminoglycan
HYP: hydroxyproline
IDD: intervertebral disc degeneration
N-CDH: N-cadherin
NP: nucleus pulposus
PG: proteoglycan
IOD: integral optical density
RT-PCR: reverse transcription-polymerase chain reaction
